# Management of Cervical Kyphotic Deformity Associated With Loeys-Dietz Vasculopathy and Cardiac Transplantation: Case Report, Literature Review, and Strategies for Complex Skeletal Dysplasias

**DOI:** 10.7759/cureus.20503

**Published:** 2021-12-18

**Authors:** Daniel A Donoho, Timothy G Singer, Tyler Lazaro, David F Bauer

**Affiliations:** 1 Pediatric Neurosurgery, Children's National Hospital, Washington, USA; 2 Surgery, University of California Los Angeles David Geffen School of Medicine, Los Angeles, USA; 3 Pediatric Neurosurgery, Texas Children's Hospital, Houston, USA

**Keywords:** cervical kyphosis, loeys-dietz syndrome, connective tissue disorder, deformity, spine

## Abstract

Seventy-six percent of pediatric patients with Loeys-Dietz syndrome (LDS), a connective tissue disorder driven by a transforming growth factor-beta (TGF-B) pathway mutation, manifest cervical spine malformations. A prior series showed that 16% required surgical stabilization. Spine surgery in LDS is associated with an 88% complication rate due to poor bone quality and cerebrovascular ectasia.

Of 77 patients with LDS, one patient who required spine surgery was identified in an institutional database from 2010 to 2020. A 15-year-old with LDS presented with symptomatic cervical myelopathy from a rapidly progressive and unstable cervical deformity. We performed a C5-6 corpectomy and an O-T2 posterior spinal fusion with recombinant human bone morphogenetic protein-2 (rhBMP-2). We achieved correction of her kyphosis and normalization of her neurologic status. She is neurologically well one year postoperatively with bony fusion.

The management of a pediatric patient with LDS, orthotopic heart transplantation (OHT), and craniocervical deformity with instability is a novel challenge. Long-segment constructs are beneficial, rather than sparing the occiput or cervicothoracic junction. Off-label BMP may aid an LDS patient with TGF-B mutation and sternotomy. Surgeons should continue immunomodulatory and antiplatelet medications when required for OHT.

## Introduction

Loeys-Dietz syndrome (LDS) is a rare connective tissue disorder associated with transforming growth factor-beta receptor 1 (TGFBR-1) and transforming growth factor-beta receptor 2 (TGFBR-2) mutations [1]. Patients with LDS have severe skeletal dysplasias, osteoporosis, and fragility fractures [2]. The previous series have shown that 76% of LDS patients have cervical spine abnormalities and 16% require surgery for cervical stabilization [3]. Because our institutional experience is at a quaternary center with strong cardiac surgery referrals, just one patient out of 77 with LDS was identified as requiring surgery. Spine surgery in LDS is high-risk; in the only case series, seven of eight patients required re-operation for complications. Complications were primarily due to symptomatic pseudoarthrosis and instability [3] in the setting of vascular ectasias and anatomic abnormalities. We describe our avoidance of these complications in a 15-year-old girl with LDS causing cervical deformity and myelopathy.

## Case presentation

This 15-year-old female came to care at six years of age with a 6 cm aortic root aneurysm. She had multiple tortuous vessels and a TGFBR-1 mutation in exon 4 (c.797A>G) [4] and was diagnosed with LDS. She underwent a complex aortic root reconstruction, including aortic valve replacement, complicated by heart failure requiring orthotopic heart transplantation (OHT) and recurrent aneurysm requiring revision aortic arch reconstruction. Heart failure and aneurysm recurrence ensued due to the Loeys-Dietz vasculopathy. She had normal cognitive development and normal neurological function until the present episode.

One year after her heart transplant, she was observed to have scoliosis on standing and underwent spine imaging. She had mild thoracic levoscoliosis without cervical kyphosis (Figure 1A). She had no thoracolumbar progression from age 7 to 13 years but developed cervical kyphosis (Figure 1B), with associated painful C5-6 spondylolisthesis (grade 2 anteriolisthesis; Figure 1C), and she presented for neurosurgical consultation. She was being evaluated for surgery when she experienced subacute quadriparesis without inciting events or trauma. She came to the emergency department with two days of bilateral symmetric weakness in her deltoids (4/5), biceps (4/5), triceps (3/5), hand intrinsic and grip (2/5), and lower extremities (4/5). She had upgoing toes and hyperreflexia in her legs. Magnetic resonance imaging of her cervical spine (Figure 1D) revealed worsening kyphosis with anteriolithesis at C5-6, causing severe spinal cord compression and new occipital-cervical instability.

**Figure 1:** Spine imaging of patient showing (A) normal alignment without cervical kyphosis, (B) developed cervical kyphosis, (C) C5-6 spondylolisthesis (grade 2 anteriolisthesis), and (D) worsening kyphosis with anteriolithesis at C5-6 with severe spinal cord compression and new occipital-cervical instability.

We performed an anterior-posterior reconstruction. The first stage was a C5-6 anterior cervical corpectomy using an expandable cage with adjustable endcaps and C4-7 plating. We then performed an occiput-T2 posterior spinal fusion. Hypoplastic lateral masses, ectatic vertebral arteries, and poor bone density led us to design a longer pedicle-screw-based construct. We placed recombinant human bone morphogenetic protein-2 (rhBMP-2) posterior-laterally for augmentation. She was placed in a cervical collar and continued her aspirin and antirejection medications (mycophenolate, tacrolimus) with meticulous surveillance of her levels.

Her immediate postoperative films showed decompression and good alignment (Figure 2A). After surgery, she returned to her neurologic baseline with a complete recovery. At her three-month follow-up (Figure 2B), nine-month follow-up (Figure 2C), and one-year follow-up (Figure 2D), she exhibited fusion without complications.

**Figure 2:** Postoperative films (A) immediately, (B) three months, (C) nine months, and (D) one year after surgery, demonstrating fusion without complications.

## Discussion

We report the results of a surgical strategy for addressing complex cervical deformity in a pediatric patient with LDS and an orthotopic heart transplant on antirejection medicine. Spinal deformity caused by skeletal dysplasias may become more common as medical care for previously fatal diseases improves.

Patients with LDS have a mercurial phenotype. Although sternotomy during infancy [5] or childhood [6] is associated with spinal deformity, our patient was stable for five years until she had rapidly progressive deformity and instability. Axial growth and skeletal maturation may play a role. We recommend yearly standing full-length scoliosis films with dynamic spot films focusing on two areas of interest in LDS: the lumbosacral junction and the cervical spine. Similarly, since we found rapidly progressive aneurysmal disease of the carotids during interval follow-up, vascular imaging such as computed tomography angiogram could be performed immediately before surgery.

Although spine surgery in LDS is treacherous [3], we achieved bony fusion using anterior corpectomy, posterior long segment pedicle screw anchors, and BMP. Anterior reconstruction using an adjustable cage minimizes endplate violations and permits customization of the deformity correction. Posterior stabilization required many potential segments since her dysplasia prevented cannulation of the pedicles and lateral masses at multiple levels. Although one lateral mass screw pulled out, the construct exhibited bony fusion at one year.

We use BMP sparingly to reduce the likelihood of spinal canal compromise or neurovascular compression [7], placing BMP into the posterior-lateral bony surfaces, facet joints, or spanning the posterior elements. Although rhBMP-2 is osteogenic, osteoconductive, and osteoinductive in vivo, interaction with the mutated TGFBR-1 pathway is unknown. In pediatric patients, rhBMP-2 is used off-label with informed consent from the family. rhBMP-2 has an established adverse effect profile including malignancy, heterotopic ossification, and wound complications; we avoid it for anterior surgery [8]. In adults, rhBMP-2 may increase the risk of malignancies [9]. Mutations in the TGFBR superfamily (such as LDS) also increase the risk of malignancy [10]. In our institution's series of rhBMP-2 uses in pediatric patients, we have not observed a case of pediatric malignancy [11].

Connective tissue disorders can cause heart failure requiring transplantation due to vascular abnormalities [12]. Although we have little prior data on pediatric patients after cardiac transplant, solid organ transplant patients requiring spinal fusion had more complications and were four times more likely to die within one year of surgery compared to controls [13]. Adults undergoing cervical fusion after transplant are at high risk of complications and death [13,14], but only one pediatric report exists [15].

We continue immunomodulatory medications and aspirin through surgery. Stopping immunomodulatory medications for spine surgery can cause organ rejection [16], but these medications may harm bone health [17] and inhibit fusion. Our patient was receiving tacrolimus, which is associated with post-transplant osteoporosis [18], though in vivo studies suggest tacrolimus (FK506) may be less harmful [19] and may even promote osteogenesis. In a rodent model, tacrolimus does not interfere with rhBMP-2 and promotes bony healing when rodents receive adenovirally-transduced rhBMP-2-expressing mesenchymal stem cells [20]. Accordingly, it is reasonable to use rhBMP-2 in patients receiving tacrolimus for immunomodulation. We achieved excellent bony fusion while maintaining therapeutic levels of tacrolimus and mycophenolate mofetil.

## Conclusions

Pediatric patients with morbid connective tissue disorders may benefit from comprehensive surgical approaches to spinal deformity. We present the first report of a patient with LDS status post-OHT requiring cervical deformity correction. Although prior series implicated a catastrophic failure rate in LDS patients, we achieved neurologic recovery and bony fusion after anterior-posterior reconstruction with corpectomy and plating, followed by long-segment fixation from the occiput to multilevel cervicothoracic pedicle screws with off-label use of BMP supplementation.
